# Frequency-Modulated Continuous Wave Radar Respiratory Pattern Detection Technology Based on Multifeature

**DOI:** 10.1155/2021/9376662

**Published:** 2021-08-09

**Authors:** Qisong Wang, Zhening Dong, Dan Liu, Tianao Cao, Meiyan Zhang, Runqiao Liu, Xiaocong Zhong, Jinwei Sun

**Affiliations:** School of Instrumentation Science and Engineering, Harbin Institute of Technology, Harbin, Heilongjiang 15001, China

## Abstract

Respiratory diseases including apnea are often accompanied by abnormal respiratory depth, frequency, and rhythm. If different abnormal respiratory patterns can be detected and recorded, with their depth, frequency, and rhythm analyzed, the detection and diagnosis of respiratory diseases can be achieved. High-frequency millimeter-wave radar (76–81 GHz) has low environmental impact, high accuracy, and small volume, which is more suitable for respiratory signal detection and recognition compared with other contact equipment. In this paper, the experimental platform of frequency-modulated continuous wave (FMCW) radar was built at first, realizing the noncontact measurement of vital signs. Secondly, the energy intensity and threshold of respiration signal during each period were calculated by using the rectangular window, and the accurate judgment of apnea was realized via numerical comparison. Thirdly, the features of respiratory and heart rate signals, the number of peaks and valleys, the difference between peaks and valleys, the average and the standard deviation of normalized short-term energy, and the average and the standard deviation and the minimum of instantaneous frequency, were extracted and analyzed. Finally, support vector machine (SVM) and K-nearest neighbor (KNN) were used to classify the extracted features, and the accuracy was 98.25% and 88.75%, respectively. The classification and recognition of respiratory patterns have been successfully realized.

## 1. Introduction

According to the World Health Organization, 27% of the world's population is suffering from respiratory problems, and 2%–7% of adults have obstructive sleep apnea [1]. Apnea can pose a threat to people's life, and chronic respiratory diseases can also affect people's health subtly [2, 3]. Therefore, the research on the classification of apnea and abnormal respiratory patterns is of great significance to the protection of life and health. At present, the more advanced contact vital signal detection methods include Forcecardiography [4], Seismocardiography [5], Gyrocardiography [6, 7], and Piezoresistive Breathing Sensing System [8, 9] with wearable shell for measuring respiration. Advanced noncontact detection equipment includes remote wireless monitoring system [10, 11], millimeter-wave radar system [12] for detecting multiple vital signs, active integrated antenna and envelope detector [13, 14], monitoring system integrated into hearing protection device [15] for detecting heartbeat and pulse, etc. High-frequency millimeter-wave radar has the advantages of small size, low power consumption, and high accuracy [16]. It can detect the movement as small as a few millimeters, so it can be used to measure the microvibration of respiration and heartbeat [17].

Recently, Petkie et al. [18] proposed a heterodyne radar system for remote measurement of respiration and heart rate, which could measure respiration and heart rate within 50 meters. Bakhtiari et al. [19] developed a compact millimeter-wave sensor for remote detection of human vital signs (respiration and heart rate). The system could be applied to a wide range of isolation sensing, including patient health care, biological measurement, and general remote vibration measurement. Kao et al. [20] adopted fully integrated Doppler miniature radar for noncontact vital signs and vibration detection using smaller wavelength to achieve a highly compact system for portable devices. Vinci et al. [21] proposed a novel remote respiratory and heartbeat monitoring sensor based on a single-base radar based on a six-port interferometer, operating at 24 GHz. The advantages of the six-port receiver are high-range measurement accuracy on the micron scale and low system complexity. Wang et al. [22] focused on the development of linear frequency modulation continuous wave (LFMCW) radar for noncontact range tracking of vital signs such as respiration signal and presented an algorithm of distance tracking based on phase. Yang et al. [23] took advantage of 60 GHz millimeter wave in sleep testing for vital signs. The system was able to monitor the respiration and heartbeat and recognize the sleep posture.

Although some progresses in the respiration detection based on millimeter-wave radar have been made, most of the frequency ranges used in millimeter-wave radar belong to low frequency such as 24 GHz and 35 GHz [24, 25]. And the measurement accuracy is always low. In addition, the majority of the millimeter-wave radar systems are with large sizes [26]. Without miniaturization and portability, the practicability will be restricted to a large extent in many aspects such as home and medical institutions. Besides, the radar signals always contain a variety of contamination, reducing the signal-noise-ratio (SNR) and the accuracy of respiration and heart rate measurement. And the current abnormal respiratory patterns are able to be detected only. However, there is no further classification [27].

To address the problem, this paper builds a noncontact vital signal-detecting system based on frequency-modulated continuous wave (FMCW) radar to realize the estimation of human micromotion parameter. By capturing the reflected signal, the FMCW radar system could obtain the distance, speed, and angle of the measured object [28]. Then, the respiration and heart rate were distinguished through calculating the vibration amplitude and frequency.

In terms of apnea judgment, we combined respiration signal and heart rate signal to do the joint apnea judgment. The rectangular window was selected to segment the vital signal. Then, the energy intensity and threshold of each segment were calculated. Next, the judgment result was output after comparing the energy intensity and the threshold.

In accordance with recognition of different respiratory patterns, experiments of 5 kinds of respiratory patterns, such as normal respiration, Biot's respiration, tachypnea, bradypnea and Cheyne–Stokes respiration, were designed and conducted separately [29]. The preprocessing and feature extraction were carried out afterwards: the valley to peak difference (VPD) peak-finding was utilized to extract the peak value, the valley value, and the difference between them [30]. After calculating the average and standard deviation of the normalized short-term energy [31], Hilbert–Huang transform (HHT) was taken advantage of to extract the average, standard deviation, and minimum of the instantaneous frequency [32]. Finally, we used support vector machine (SVM) and K-nearest neighbor (KNN) algorithm to do the classification, realizing the recognition of different respiratory patterns successfully.

The structure of the paper is as follows: Section 2 introduces the FMCW radar-based experimental platform and the data acquisition.  Section 3 describes the data acquisition and processing.  Section 4 illustrates the apnea judgment through energy intensity and threshold.  Section 5 represents the respiratory pattern classification. In Section 6, the research contents of this paper are discussed and compared with other research studies in this field.  Section 7 summarizes this paper.

## 2. Data Acquisition Based on FMCW Radar Experimental Platform

The schematic diagram of the vital signal-detecting system based on FMCW radar is shown in Figure 1. Initially, a synthesizer generates a linear frequency modulation (LFM) (whose frequency is linear with time) pulse, which is emitted by the transmit antenna (TX antenna). After reaching the measured object, the reflected pulse is captured by the receive antenna (RX antenna). The mixer combines the RX and TX signals and generates an intermediate frequency (IF) signal. The instantaneous frequency of the output IF signal is equal to the difference of the instantaneous frequency of the two signals. The phase of the output IF signal is equal to the difference of the phase of the two signals. After being bandpass filtered and sampled by analogue-to-digital converser (ADC), the sampling rate of ADC is 2 MHz, and the ADC resolution is 10 bit. The data are packaged by the processor. From USB to serial port, the acquired data are sent to the PC. Subsequently, with data processing including fast Fourier transform (FFT), the waveform and frequency of the vital signals of respiration and heart rate are gained.

The experiment platform is composed of millimeter-wave sensor (IWR1642 (Texas Instruments, America)), microcontroller (TM4C1294NCPDT (Texas Instruments, America)), FLASH memory, and power circuit. The hardware block diagram is implied in Figure 1. The power circuit includes the following:

- Power management chip, LP87524 (Texas Instruments, America), converts the externally input voltage (5 V) into the voltage required (1.2 V, 1.3 V, 1.8 V, and 3.3 V) by the millimeter-wave sensor, which needs to be controlled through I2C compatible serial interface and enable signal.
- Circuit protection chip, TPD4E004 (Texas Instruments, America), is used for interference suppression and electrostatic protection.
- Linear regulator, BL9193 (Belling, China), converts the input voltage, 5 V, to 3.3 V for the microcontroller.

The millimeter-wave sensor, IWR1642, communicates with the FLASH memory through Queued Serial Peripheral Interface (QSPI) to realize the data reading and erasing. The microcontroller can achieve the programming in the integrated digital signal processing (DSP) subsystem of the millimeter-wave sensor through the JTAG interface. The collected signals are converted by the microcontroller and sent to the PC via USB for data processing.  Figure 2 shows the experimental platform of the millimeter-wave radar. The actual power of the millimeter-wave radar experimental platform is 3.6 W.

The distance resolution *d*_res_ and speed resolution Δ*ω* of the system are determined by the bandwidth and sweep frequency, respectively. The specific formula is shown as follows:

(1) $$\begin{array}{c} d_{\text{res}}=\frac{c}{2B}, \end{array}$$

(2) $$\begin{array}{c} \Delta \omega =\frac{2\pi }{N}. \end{array}$$

In order to enhance the FMCW radar parameter resolution, combined with the IWR1642, the linear frequency modulation parameters for radar measurement are set in Table 1.

### 2.1. Bandwidth

The bandwidth needs to be increased proportionally. Therefore, the maximum continuous bandwidth, 4 GHz, in which the millimeter-wave sensor IWR1642 could support, was chosen in order to improve the distance resolution.

### 2.2. Number of Sweep Frequency (*N*)

The number of sweep frequencies needs to be enhanced. However, increasing the number of sweep frequency will lead to longer processing time. Considering the speed resolution and algorithm efficiency comprehensively, the number of sweep frequency of each linear FM frame was 100.

### 2.3. Duration of Sweep Duration (*T*_*c*_)

The bandwidth of the radar measurement is related to the duration of frequency sweep. The duration of sweep frequency was set to 50 *μ*s so as to ensure the maximum bandwidth of the radar.

For the other parameters, the initial frequency *F*_*c*_ = 77 GHz, the slow time axis sampling frequency *F*_*s*_ = 20 Hz, and the fast time axis sampling frequency *F*_*s*_∼_fast_ = 2 MHz were defined.

## 3. Data Acquisition and Processing

There were 20 healthy subjects with an average age of 24. Before the experiment, each person sat in front of the test radar into a calm state and then began the formal measurement. Each simulated respiration method is shown in Table 2. The number of apnea simulations was 5 for each person, which formed 100 samples in total. Each respiratory pattern was simulated 8 times for each person, forming 160 samples of each respiratory pattern, and there were 800 samples in total.

Adults breathe about 16–20 times per minute normally. Biot's respiration belongs to a pathological periodic respiration: one or more strong breaths are followed by a long breath stop, and then several strong breaths arise again, with a cycle of 10–60 seconds [33]. Tachypnea forms when the respiratory frequency of adults is more than 20 times per minute. Bradypnea means that the respiratory rhythm is regular, but the frequency is less than 10 times per minute. Cheyne–Stokes respiration happens along with the gradual weakening of respiration, so that the respiration stop and the gradual increase appear alternately, showing a tidal wave-like trend [34]. The waveforms of the five respiratory patterns are indicated in Figure 3.

Subjects were simulated with apnea and five respiratory patterns (normal respiration, Biot's respiration, tachypnea, bradypnea, and Cheyne–Stokes respiration). The number of apnea simulations was 5 for each person, which formed 100 samples in total. Each respiratory pattern was simulated 8 times for each person, forming 160 samples of each respiratory pattern, and there were 800 samples in total.

### 3.1. Experiment of Optimum Measurement Distance

In order to find out the best measurement distance of the FMCW radar, three distance experiments were carried out. The FMCW radar was 10 cm, 30 cm, and 50 cm away from the chest, respectively, and the data were collected for 1 min in each experiment. The number of frames of the collected data was recorded. When using FMCW radar for data acquisition, due to external or internal interference, data loss will often occur, leading to the mutation of the corresponding point of that frame. If there was a mutation in the corresponding point, the data of this frame got lost. Therefore, the quality of the collected data could be judged according to the number of mutations.

The frames and waveforms corresponding to the data collected by millimeter-wave radar at 10 cm, 30 cm, and 50 cm are shown in Figure 4 respectively.

We conducted experiments on 20 subjects at 10 cm, 30 cm, and 50 cm, respectively, and recorded their mutation points. The recorded results are shown in Table 3.

By comparison, when the experimental distance is 30 cm, the data corresponding to the frame have fewer mutation points and higher accuracy.

### 3.2. Separation of Vital Signal Based on Bandpass Filter

After data acquisition, it is necessary to extract and separate the respiration and heart rate signals from the microdisplacement vibration of the raw signals. Phase difference signal refers to the phase difference part of the IF signal, which includes the respiration and heartbeat information of the human body.  Figure 5 illustrates the separation process of the vital signals of respiration and heart rate. Both respiration and heart rate cause weak vibrations on the body surface. The frequency of the vibration from respiration is 0.1–0.6 Hz [35], and the amplitude is 1–12 mm. The frequency of vibration from heartbeat is 0.8–4.0 Hz [36], and the amplitude is 0.1–0.5 mm. In view of the difference in the amplitude and frequency of body surface vibration caused by respiration and heart rate, bandpass filters with different frequencies can be applied [37]. The specific process is as follows:

1. Perform the distance FFT on the data collected by millimeter-wave radar.
2. Extract the phase from the selected range bin and unwrap the phase.
3. Apply the bandpass filter to the phase different signal. When the frequency band is 0.1–0.6 Hz, the respiratory signal is obtained. When the frequency band is 0.8–4.0 Hz, the heart rate signal is got.

After separating the respiratory and heart rate signals, the frequencies were calculated. The spectrum estimation of respiratory signal based on FFT and peak interval was performed [38]. The final respiratory rate was output under the confidence degree. Because the measurement of heart rate is based on the distance difference between the tiny movement of heart contraction and diastole, and the phase change caused by the difference, according to the micro-Doppler principle, when the human body appears, a large-scale movement will affect its accuracy. Therefore, it was a need to determine whether the segment was damaged. The undamaged data were put into the valid value buffer while the data whose energy exceeded the threshold were abandoned. Then, the spectrum estimation based on FFT, autocorrelation, and peak interval was performed, and the confidence degrees of them were calculated. Similarly, the final heartbeat frequency was output with the decision based on the confidence degree.

### 3.3. Reliability Verification of Millimeter-Wave Radar Measurement Method

While respiration was measured by the millimeter-wave radar, a respiratory belt (RSB-EQ001 (ADInstruments, Australia)) was used to record respiratory rate. The error was calculated to obtain the reliability of the system. The experimental data are shown in Table 4.

Through observation, the maximum error of respiratory rate measured by millimeter-wave radar is 6.67%, so the measurement results are accurate. The respiration measurement by the millimeter-wave radar method is reliable.

While using millimeter-wave radar to measure the heart rate, the oximetry (YX303 (Yuwell, China)) was used to record the heart rate. The experimental data are shown in Table 5.

Through observation, the maximum error of heart rate measured by millimeter-wave radar is 2.90%, so the measurement results are accurate. It is reliable to measure heartbeat by millimeter-wave radar.

### 3.4. Frame Data Processing

When using FMCW radar for data acquisition, due to external or internal interference, data loss of a certain frame will often occur, leading to the mutation of the corresponding point of that frame, as shown in Figure 6.

The lost data have a certain impact on the results, so the data should be processed. This paper proposed two processing methods, and the results of the two processing methods (apnea judgment) were compared as shown in Figure 7:

- Remove the mutation points.
- Add an average value to the point where there is a mutation: for example, if there is mutation at the 15th point, add an average value of the 15th and 16th points between the 15th and 16th points.

There was a small period of misjudgment for apnea by method 1, and no misjudgment by method 2. Method 2 has better processing effect on abnormal data, so method 2 is chosen to process abnormal data.

## 4. Judgment of Apnea Based on Energy Intensity and Threshold

### 4.1. Energy Intensity and Threshold Judgment

The respiration and heart rate signals belong to nonperiodic deterministic signals, which can be illustrated by energy intensity. The energy intensity of the discrete signal is expressed as follows:

(3) $$\begin{array}{c} E\left(i\right)=\sum_{-\infty }^{\infty }{\left|x\left(i\right)\right|}^{2}, \end{array}$$

where *i* represents the position of discrete signal points, *E*(*i*) represents the energy intensity, and *x*(*i*) represents the discrete signal. The energy intensity reflects the magnitude of the respiration and heart rate signals. Hence, the signal threshold is set to do the comparison: when the energy intensity value of the vital signal reduced by more than 50% compared with normal respiration, the apnea occurred. The threshold, *D*(*n*), was divided into three sections, as shown below. The energy intensity will be higher than the threshold during normal respiration, and that is lower than the threshold during apnea:

(4) $$\begin{array}{c} n=1:D\left(n\right)=E\left(1\right)\times 50\%,\\ 2\leq n<5:D\left(n\right)=\frac{\sum_{i=n-4}^{i=n}E\left(i\right)}{n}\times 50\%,\\ n\geq 5:D\left(n\right)=\frac{\sum_{i=n-4}^{i=n}E\left(i\right)}{5}\times 50\%, \end{array}$$

where ∑_*i*=*n*−4_^*i*=*n*^*E*(*i*) is on behalf of the energy intensity in the front *n* segments. When *n*=1, the signal threshold is 50% of its energy intensity; when 2 ≤ *n* < 5, the signal threshold is 50% of the average value of *n*-segment signal energy intensity; when *n* ≥ 5, the signal threshold is 50% of the average value of the energy intensity of the first 5 signals after the two signals.

### 4.2. Apnea Test Verification

The energy intensity and threshold were taken advantage of to judge the apnea: in the beginning, the rectangular window was used to segment the respiratory signals and heart rate signals, and the energy intensity and threshold of each segment were calculated. When the energy intensity was higher than the threshold during normal respiration, “0” was output. During apnea, the energy intensity was lower than the threshold and “1” was output. The subjects were required to simulate the respiratory pattern of “normal respiration-apnea-normal respiration,” and Figure 8 indicates the judgment results.

For respiratory signal, actual apnea started at 84th point and stopped at 145th point. The results of apnea judgment based on respiratory signals showed that it started from the 90th point and stopped at the 143rd point, with a detecting accuracy of 86.9%.

For heart rate signal, actual apnea started at 83rd point and stopped at 139th point. The results of apnea judgment based on heart rate signal showed that it started at the 92nd point and stopped at the 138th point, and the monitoring accuracy was 82.1%.

It can be found that the respiratory signal and heart rate signals can distinguish the apnea with the energy intensity and threshold. The judgment accuracy of the respiratory signal is higher than that of the heart rate signal, but the heart rate signal can also play a role in assisting judgment. Thus, not only can the judgment of apnea rely on breathing, but also heart rate can be used as a reference.

## 5. Classification of Respiratory Pattern Based on Multifeature Extraction and Machine Learning

Chronic respiratory diseases are also detrimental to people's health, so it is indispensable to judge the chronic respiratory diseases. Respiratory diseases are often accompanied by abnormal respiratory depth, frequency, and rhythm. Different combinations of them often result in different abnormal respiratory patterns [39]. For example, excessive respiratory frequency will lead to tachypnea. Abnormal respiratory rhythms will provoke Cheyne–Stokes respiration likewise. We mainly focus on five respiratory patterns: normal respiration, Biot's respiration, tachypnea, bradypnea, and Cheyne–Stokes respiration.

### 5.1. Feature Extraction of Respiratory Pattern

#### 5.1.1. The Number of Peaks, the Number of Valleys, and the Difference between Them

The vital signal processing usually involves peak detection and peak interval searching. Peak detection aims at finding the position and amplitude of the local maximum in certain signal. We chose the VPD peak-finding algorithm [30], which eliminated all false peaks induced by noise through iteration, until the results of the number of peaks in two consecutive iterations were consistent. The program block diagram is implied as follows in Figure 9, and the steps are as follows:

(a) *Preprocessing*. Use a three-point moving average smoothing filter to improve the SNR. Next, apply filters forward and backward to remove any phase shifts resulting from filtering.
(b) *Maximum and Minimum Detection*. Detect all the peaks and valleys in the signal and determine their positions.
(c) *Judgment of Peak Point and Valley Point Position*. Compare the positions of the first peak point and the first valley point under the condition that VPD processing starts at the valley. If the peak point appears first, discard it, and start acquiring the signal from the first valley point. Consequently, there are not corresponding valley points along with discarded peak points.
(d) *Calculation of the Difference between Peak and Valley*. VPD is expressed in equation (5), and the algorithm will search for certain condition in the VPD series, as given in (6). Instances meeting this condition are considered to be over-detected, so the corresponding peak points and peak positions are deleted from the candidate sequence:
  (5) $$\begin{array}{c} \text{VPD}\left(k\right)=P\left(k\right)-V\left(k\right),\;k=1,2,3,\ldots ,m, \end{array}$$
  (6) $$\begin{array}{c} \text{VPD}\left(k\right)<0.7*\frac{\left\{\text{VPD}\left(k-1\right)+\text{VPD}\left(k\right)+\text{VPD}\left(k+1\right)\right\}}{3}. \end{array}$$
(e) *Repeated VPD Processing*. Repeat VPD processing until the number of peak points in two consecutive iterations maintains unchanged, so that all peaks provoked by noise and artifacts can be eliminated.

In the experiment, the number of peaks, the number of valleys, and the difference between them of the five respiratory patterns were selected as the features. In the light of the characteristics of the respiratory patterns, the subjects simulated different respiratory patterns. For each pattern, 80 datasets were collected as training samples. The number of peaks and valleys and the difference between them were recorded in 1 minute. The millimeter-wave radar sampled 20 points per second, namely, about 1200 points per minute. A set of samples with peak value in each pattern are demonstrated in Figure 10, and the recorded data (part) are listed in Table 6.

As can be seen from Table 6, the number of peaks, the number of valleys, and the difference between them vary in different respiratory patterns. For example, a statistical analysis of all the samples showed that the average number of peaks of respiratory tachypnea per minute was 20.15, and the average number of peaks of respiratory bradypnea was 14.87. At the same time, the difference between the peak and valley points of tachypnea is smaller than that of bradypnea.

Later, we compared the VPD peak-finding algorithm with the common peak-finding function, findpeaks. Taking normal respiration as an example, the peak and valley points obtained by the findpeaks function are displayed in Figure 11. In the same way, we recorded 80 sets of training samples for each respiratory pattern gained by the findpeaks function for 1 minute, respectively.  Table 7 implies the recorded data (part).

It can be seen that the peak points are not screened, which increases the number of peak points dramatically. At the same time, the number of peak points and valley points is equal. In this paper, we used the number of peaks, the number of valleys, and the difference between them as the feature. Consequently, we use the VPD peak-finding algorithm for feature extraction.

#### 5.1.2. Normalized Short-Term Energy Average and Standard Deviation

Since the energy of the respiratory signal changes with time, there is a certain energy difference between weak respiratory and strong respiratory. Thus, analyzing the short-term energy of the respiratory signal is able to describe the characteristic change of respiration. Normalization can map the data to [−1, 1] to remove the amplitude difference of respiratory signals among different subjects and different respiratory patterns. The normalization is expressed as follows:

(7) $$\begin{array}{c} x=\frac{x_{0}}{{\left|x_{0}\right|}_{\max}}, \end{array}$$

where |*x*_0_|_max_ is the maximum in the absolute value of the raw respiratory signal amplitude. After normalization, the respiratory signal is defined as follows:

(8) xn=−1+x−xminx−maxxmin·2,

where *x*_max_ and *x*_min_ are the maximum and minimum of the respiratory signal amplitude after normalization.

The short-term energy of the respiratory signal is defined as follows:

(9) $$\begin{array}{c} E_{n}={\sum_{m=-\infty }^{+\infty }\left[x_{n}\left(m\right)w\left(n-m\right)\right]}^{2}={\sum_{m=n-\left(N-1\right)}^{n}\left[x_{n}\left(m\right)w\left(n-m\right)\right]}^{2}, \end{array}$$

where *w*(*n*) is the window function, *N* is the window length, and windowing is capable of reducing the truncation effect of the respiratory frame. When the window function is a rectangular window, equation (11) turns to

(10) $$\begin{array}{c} E_{n}=\sum_{m=n-\left(N-1\right)}^{n}x_{n}{}^{2}\left(m\right). \end{array}$$

We applied a rectangular window whose length is 4 seconds, and millimeter-wave radar samples 20 points per second (80 points in 4 seconds), that is, *N* = 80. The applied rectangular window is written as

(11) $$\begin{array}{c} w\left(n\right)=\left\{\begin{array}{cc} 1, & 0\leq n<N-1,\\ 0, & \text{other}. \end{array}\right. \end{array}$$

Subjects simulated different respiratory patterns, and the normalized short-term energy was calculated from the collected data. 80 datasets were collected for each pattern as training samples, and a set of data was opted from each respiratory pattern sample to perform normalized short-term energy calculation. The results are manifested in Figure 12.

It is undeniable that the short-term energy during tachypnea exceeds that of bradypnea, and the short-term energy during apnea is almost zero. Additionally, normal respiration, tachypnea, and tachypnea maintain the same respiratory intensity basically, and the short-term energy changes slightly. The intensity of Biot's respiration decreases first and then rises. The intensity of Cheyne–Stokes respiration soars initially and drops later. The short-term energy change of Biot's and Cheyne–Stokes respiration is greater. In expectation of observing the amplitude and the trend, the average and standard deviation of the short-term energy (part) of the 5 respiratory patterns were calculated separately and are given in Table 8.

#### 5.1.3. The Average Value, Standard Deviation, and Minimum of Instantaneous Frequency

The instantaneous frequency represents the transient frequency characteristics of the signal at local time points, and the instantaneous frequency over the entire duration reflects the time-dependent law of the signal frequency. For signal *X*(*t*), the Hilbert transform can be used to obtain *Y*(*t*), as demonstrated in the following equation:

(12) $$\begin{array}{c} Y\left(t\right)=\frac{1}{\pi }PV\left(\int_{-\infty }^{\infty }\frac{X\left(\tau \right)}{t-\tau }\text{d}\tau \right), \end{array}$$

where *PV* is the Cauchy principal value. *Y*(*t*) is the convolution of *X*(*t*) and (1/*πτ*). As a result, *X*(*t*) and *Y*(*t*) form a conjugate complex pair, so an analytical signal *Z*(*t*) can be got in equation (13), where *a*(*t*) and *θ*(*t*) are on behalf of the amplitude and phase:

(13) $$\begin{array}{c} Z\left(t\right)=X\left(t\right)+iY\left(t\right)=a\left(t\right)e^{i\theta \left(t\right)}, \end{array}$$

(14) $$\begin{array}{c} a\left(t\right)={\left[X^{2}\left(t\right)+Y^{2}\left(t\right)\right]}^{\left(1/2\right)}, \end{array}$$

(15) $$\begin{array}{c} \theta \left(t\right)=\mathrm{arc}\text{ tan}\left(\frac{Y\left(t\right)}{X\left(t\right)}\right). \end{array}$$

There are many ways to define the imaginary part. However, the Hilbert transform provides a unique imaginary part, which forms an analytic function. Once the phase is obtained, the instantaneous frequency can be got because the instantaneous frequency is the derivative of phase:

(16) $$\begin{array}{c} \omega =\frac{\text{d}\theta \left(t\right)}{\text{d}t}. \end{array}$$

The subjects simulated different respiratory patterns. Data were collected, and HHT was performed. Taking a dataset of Biot's respiration as an example, the raw waveform and instantaneous frequency are shown in Figure 13.

It is evident that in Biot's respiration, the instantaneous frequency during normal respiration period is significantly higher than that during the apnea period, and the instantaneous frequency of the apnea is almost zero. In this case, we inferred that the instantaneous frequency of strong respiration is higher than that of weak respiration. To verify this, one experimental dataset of tachypnea and bradypnea was taken out, and HHT was done.  Figure 14 gives information about the instantaneous frequency. Since the instantaneous frequency of apnea in Biot's respiration was nearly 0, we implied that the instantaneous frequency of apnea in Cheyne–Stokes respiration was nearly 0 as well. Equally, one experimental dataset of normal and Cheyne–Stokes respiration was taken out separately, and HHT was operated so as to get the instantaneous frequency. The result is indicated in Figure 15.

It is obvious that the instantaneous frequency of tachypnea is higher than that of bradypnea. And the tachypnea and bradypnea maintained the same intensity basically, with small changes in the instantaneous frequency. The respiratory intensity of Biot's respiration first declines and then leaps. The instantaneous frequency changes dramatically, and the instantaneous frequency is almost zero during apnea. For the purpose of observing the amplitude and trend of the instantaneous frequency, we calculated the average and standard deviation of the instantaneous frequencies of 80 training samples of 5 respiratory patterns. The instantaneous frequencies of Biot's and Cheyne–Stokes respiration are 0 basically, so the minimum instantaneous frequency can be calculated to distinguish Biot's respiration and Cheyne–Stokes respiration from the other 3 respiratory patterns. The average, standard deviation, and minimum of the instantaneous frequencies (part) of the 5 respiratory patterns are listed in Table 9.

### 5.2. Classification and Experimental Verification of Respiratory Patterns Based on Machine Learning

In this paper, the KNN method and SVM method are used to classify the samples. The KNN algorithm has the advantages of simplicity, efficiency, and low cost of retraining. Because the KNN method mainly depends on the surrounding limited adjacent samples, rather than the method of discriminating the class domain to determine the category, therefore, for the sample set to be divided which has a lot of crossover or overlap of the class domain, the KNN method is more suitable than other methods. However, the classification of call pattern in this paper is just suitable for this situation, so the KNN method is selected for classification learning. At the same time, the results of SVM method have good generalizability. It can solve the machine learning problem in the case of small sample, can solve the high-dimensional problem, and can avoid the neural network structure selection and local minimum point problem. In addition, it can obtain a low error rate, and SVM can make good classification decisions for data points outside the training set [40]. Therefore, we choose the SVM method as the second classification learning method.

Firstly, we conducted the experiment of the 10-fold cross-validation method. We divided the samples into ten groups. Samples of each respiratory pattern were labeled: normal respiration (1), Biot's respiration (2), tachypnea (3), bradypnea (4), and Cheyne–Stokes respiration (5). Taking 9 groups of samples as training data and 1 group of samples as test data, the experiment was carried out in turn. The experimental results are shown in Table 10.

The average of classification accuracy of SVM is 97.88%, higher than that of KNN classification accuracy (88.75%). Next, we classify the total sample. 400 sets of data were used as training samples, and the remaining 400 sets of data were used as test samples. The confusion matrix of the two classifiers is revealed in Figure 16.

Features extracted via the VPD peak-finding algorithm, normalized short-term energy, and instantaneous frequency on all experimental data were sent into SVM and KNN classifiers for training and testing. The classification accuracy of the two classifiers is shown in Table 11.

From Table 11, the classification accuracy of SVM is 98.25%, higher than that of KNN classification accuracy (88.75%). The Cohen kappa score of SVM is 0.978125, higher than that of KNN classification accuracy (0.859375). When it comes to KNN, 21 samples of normal respiration are misjudged as Cheyne–Stokes respiration, 19 samples of Biot's respiration are misjudged as Cheyne–Stokes respiration, 4 samples of Biot's respiration are misjudged as bradypnea, and 1 sample of bradypnea is misjudged as Biot's respiration. Other two patterns, tachypnea and Cheyne–Stokes respiration, are classified correctly. When referring to SVM, 7 samples of Cheyne–Stokes respiration are misjudged as normal respiration. Other four patterns, normal respiration, Biot's respiration, tachypnea, and Cheyne–Stokes respiration, are classified correctly. The classification accuracy of tachypnea is 100%, which achieves the ideal classification.

## 6. Discussion

First of all, the FMCW radar used in this paper is a special radar technology with short wavelength electromagnetic waves. The FMCW radar can transmit signals in millimeter range. Such wavelengths are considered short wavelengths in the electromagnetic spectrum, which is one of the advantages of the technology. Another advantage of short wavelengths is high accuracy, and millimeter-wave radar systems operating at frequencies between 76 and 81 GHz (corresponding to wavelengths of about 4 mm) are able to detect movement to millimeter level. At the same time, high-frequency millimeter-wave radar has the advantages of small size, low power consumption, and high precision.

Secondly, the optimal distance for FMCW radar to obtain vital signals was found through experiments, and the respiratory and heart rate signals were separated. Meantime, abnormal data were processed. This effectively ensured that the experiments about apnea detection and the recognition of respiratory patterns related were carried out smoothly. Next, the energy intensity and threshold method were used to identify apnea.

Finally, this paper extracted three features of the five respiratory patterns: the number of peaks, the number of valleys, and the difference between them; the average and standard deviation of the normalized short-term energy; the average value, standard deviation, and minimum of the instantaneous frequency. SVM and KNN were made use of to classify the extracted features, and the accuracy rates were 98.25% and 88.75%, respectively.

According to the recorded data, the number of peaks, the number of valleys, and the difference between them have different variation trend under different respiratory patterns. For example, a statistical analysis of all the samples showed that the average number of peaks of respiratory tachypnea per minute was 20.15, and the average number of peaks of respiratory bradypnea was 14.87. At the same time, the difference between the peak and valley points of tachypnea is smaller than that of bradypnea.

Through the analysis of all the samples, the short-term energy during tachypnea exceeds that of bradypnea, and the short-term energy during apnea is almost zero. Additionally, normal respiration, tachypnea, and tachypnea maintain the same respiratory intensity basically, and the short-term energy changes slightly. The intensity of Biot's respiration decreases first and then rises. The intensity of Cheyne–Stokes respiration soars initially and drops later. The short-term energy change of Biot's and Cheyne–Stokes respiration is greater. In this paper, we used the average and standard deviation of the normalized short-term energy to describe the size and variation trend of short-term energy and took it as the second feature for the classification of respiratory patterns.

Next, we analyzed the instantaneous frequency of respiratory patterns across the entire sample. It is evident that in Biot's respiration, the instantaneous frequency during normal respiration period is significantly higher than that during the apnea period, and the instantaneous frequency of the apnea is almost zero. It is obvious that the instantaneous frequency of tachypnea is higher than that of bradypnea. And the tachypnea and bradypnea maintain the same intensity basically, with small changes in the instantaneous frequency. The respiratory intensity of Biot's respiration first declines and then leaps. The instantaneous frequency changes dramatically, and the instantaneous frequency is almost zero during apnea. Therefore, we calculated the average value, standard deviation, and minimum of the instantaneous frequency and took them as the third feature for the classification of respiratory patterns.

Finally, SVM and KNN were used for classification, and the result of SVM was obviously better than KNN. This is because SVM trains a model on the training set and then uses the model to classify the test set directly. These two steps are independent. For KNN, there is no training process. Only distance measurement is made between training data and training data to achieve classification. The accuracy of SVM and KNN is 98.25% and 88.75% separately. The proposed respiratory pattern classification method is effective and has high accuracy.

In the meantime, this paper also has some advantages in the current research field. Although there are some similar studies before [41–46], this paper has obvious advantages. For example: Nijsure et al. developed a respiratory signal monitoring system based on ultrawideband radar and proposed a point detection algorithm that distinguished normal breathing from apnea, with an accuracy rate of 81%. In this paper, the accuracy of apnea identification was higher, which was 86.9%. Lee et al. used 2.4 GHz radar to detect five respiratory patterns (dysrhythmic respiration, normal respiration, apnea, Cheyne–stokes respiration, and Cheyne–stokes variant respiration). In comparison, the FMCW wave in this paper has higher frequency, more accurate measurement, and better detection effect. Wang et al. used radar to monitor normal respiration and sleep apnea of the subjects, extracted three features of short-term mean amplitude, short-term variance, and short-term spectrum amplitude at specific points of respiratory signals, and distinguished normal respiration and apnea by pattern recognition. Additionally, the team used power and wavelet information entropy to calculate the number of sleep apnea, with the accuracy of 85% and 79%, respectively. By comparison, the accuracy of apnea detection in this paper is higher. At the same time, the classification of respiratory patterns was also carried out in addition to the judgment of apnea. Shah et al. conducted remote monitoring of patients using noninvasive radio frequency (RF) sensing to detect normal respiratory rates and abnormal breathing rates, such as elevated patterns where person experiences heavy breathing and shallow rates where minimal air is inhaled and exhaled. In the meantime, support vector machine (SVM), k-nearest neighbor (KNN), and decision tree algorithms were used to evaluate overall performance of the proposed model. We observed that the SVM classifier provided best classification accuracy (96%). Loon et al. [47] used FMCW radar to measure and identify respiratory abnormalities in patients in 2016, and accuracy was 86%. More kinds of feature are extracted in this paper, so there is a greater correlation with respiratory conditions. The detection results are better, and the accuracy rate is 98.25%.

## 7. Conclusions

With the development of medical level, no one can deny that respiratory state is closely related to human health. Thus, chronic respiratory diseases can be prediagnosed and patients will be rescued in emergency by means of detecting respiratory state in daily life. We used the FMCW radar system to detect vital signals, separated and extracted two vital signals, respiration and heart rate. We then judged apnea by way of energy intensity and threshold. The experiment of apnea under different conditions was conducted. Next, we extracted the number of peaks, the number of valleys, and the difference between them through the VPD peak-finding algorithm and compared this algorithm with the ordinary peak-finding function, findpeaks, to prove the effectiveness of the VPD algorithm. Later, we processed the respiratory signal, extracted the average and standard deviation of the normalized short-term energy, and performed HHT to extract the average value, standard deviation, and minimum of the instantaneous frequency. SVM and KNN were adopted to do the classification, and the accuracy rates were 98.25% and 88.75%, respectively, verifying the effectiveness of the extracted features and classification model.

This paper provides a noncontact, wider detection means for vital signals. Our research is expected to play a favorable role in the diagnosis of chronic respiratory diseases, provide new technologies for early respiratory diseases screening, and promote the development of millimeter-wave radar in medical fields. However, the research method of this paper also has some disadvantages. First, this study is in the laboratory stage and has not been applied to clinical trials. At the same time, the environmental requirements of radar data collection in this paper are also high, such as the impact of vibration of other objects in the room, the distance between the radar and human body, and the position relationship between the two. Our future work is applying our device to clinical trials, testing and optimizing the entire system.

## Figures and Tables

**Figure 1:** The schematic diagram and the hardware block diagram of the vital signal-detecting system based on FMCW radar.

**Figure 2:** The experimental platform of the millimeter-wave radar.

**Figure 3:** The waveforms of the five respiratory patterns: (a) normal respiration; (b) Biot's respiration; (c) tachypnea; (d) bradypnea; (e) Cheyne–Stokes respiration.

**Figure 4:** Distance experiment results: (a) frame changes during data acquisition (10 cm); (b) respiratory signal and heart rate signal waveform (10 cm); (c) frame changes during data acquisition (30 cm); (d) respiratory signal and heart rate signal waveform (30 cm); (e) frame changes during data acquisition (50 cm); (f) respiratory signal and heart rate signal waveform (50 cm).

**Figure 5:** Flowchart of separation calculation of respiration and heart rate.

**Figure 6:** Mutations in frame corresponding point lost during data acquisition.

**Figure 7:** Comparison of two processing methods: (a) signal processing by method 1; (b) signal processing by method 2.

**Figure 8:** Energy intensity, threshold, and judgment results of respiratory and heart rate signals: (a) respiratory signal; (b) heart rate signal.

**Figure 9:** The program block diagram of VPD.

**Figure 10:** Peak-finding results of 5 respiratory patterns: (a) normal respiration; (b) Biot's respiration; (c) tachypnea; (d) bradypnea; (e) Cheyne–Stokes respiration.

**Figure 11:** The result of comparison between VPD and the common peak-finding function, findpeaks.

**Figure 12:** Normalized waveforms and short-term energy of 5 respiratory patterns: (a) normal respiration; (b) Biot's respiration; (c) tachypnea; (d) bradypnea; (e) Cheyne–Stokes respiration.

**Figure 13:** The raw waveform and instantaneous frequency of Biot's respiration.

**Figure 14:** Comparison of instantaneous frequency between tachypnea and bradypnea.

**Figure 15:** Comparison of instantaneous frequency between normal and Cheyne–Stokes respiration.

**Figure 16:** The confusion matrix of different classifiers: (a) SVM; (b) KNN.

**Table 1:** The linear frequency modulation parameters for radar measurement.

Parameters	Value
*Bandwidth*	4 GHz
*N*	100
*T*_*c*_	50 *μ*s
*F*_*c*_	77 GHz
*F*_*s*_	20 Hz
*F*_*s*_∼_fast_	2 MHz

**Table 2:** Simulated respiration methods.

Respiratory patterns	Experimental methods	Experiment time (s)
Normal respiration	Normal respiration	60
Biot's respiration	Stop respire for 30 seconds and complete the respiratory cycle every 4 seconds for 30 seconds	60
Tachypnea	Complete respiratory cycle every 2 seconds for 60 seconds	60
Bradypnea	Complete respiratory cycle every 8 seconds for 60 seconds	60
Cheyne–Stokes respiration	Apnea-gradual increase in respiration-gradual decrease in respiration-apnea. Each phase is maintained for about 20 seconds	60
Apnea	Normal respire 20 seconds, apnea 20 seconds, normal respire 20 seconds	60

**Table 3:** Mutation points of different subjects at different radar distances.

Subject number	10 (cm)	30 (cm)	50 (cm)
1	9	7	13
2	8	5	10
3	10	8	13
4	9	6	12
5	9	6	12
6	8	6	11
7	11	8	13
8	9	5	13
9	8	6	12
10	9	6	12
11	10	8	14
12	11	7	12
13	9	6	13
14	8	5	10
15	8	5	11
16	9	5	12
17	10	8	13
18	9	6	12
19	9	5	14
20	8	6	12
The average	9.05	6.20	12.20

**Table 4:** A comparison of respiratory rates measured by millimeter-wave radar and respiratory belt.

Times	Millimeter-wave radar (breaths per minute (bpm))	Respiratory belt (breaths per minute (bpm))	The error (%)
1	19	20	5
2	18	19	5.26
3	16	17	5.88
4	17	18	5.56
5	22	21	4.76
6	16	15	6.67
7	20	19	5.26
8	18	19	5.26
9	20	19	5.26
10	19	20	5

**Table 5:** A comparison of heart rate measured by millimeter-wave radar and oximetry.

Times	Millimeter-wave radar (beats per minute (bpm))	Oximetry (beats per minute (bpm))	The error (%)
1	70	69	1.45
2	67	69	2.90
3	67	69	2.90
4	67	68	1.47
5	67	67	0.00
6	68	70	2.86
7	68	69	1.45
8	70	69	1.45
9	70	71	1.41
10	70	70	0

**Table 6:** Number of peaks and valleys of 5 respiratory patterns (VPD, part data).

Respiratory patterns	Number of peaks/number of valleys/difference			
Normal respiration	21/45/24	17/42/25	16/44/28	18/42/24
Biot's respiration	12/37/25	8/53/45	11/47/36	14/57/43
Tachypnea	20/38/18	22/41/19	18/41/23	24/36/12
Bradypnea	13/39/26	15/41/26	13/44/31	16/39/23
Cheyne–Stokes respiration	10/45/36	14/45/31	5/42/37	13/49/36

**Table 7:** Number of peaks and valleys of 5 respiratory patterns (the common peak-finding, part data).

Respiratory patterns	Number of peaks/number of valleys/difference			
Normal respiration	51/51/0	23/23/0	50/49/-1	45/46/1
Biot's respiration	51/50/-1	58/58/0	55/56/1	68/68/0
Tachypnea	45/45/0	49/49/0	47/46/-1	41/40/-1
Bradypnea	43/43/0	49/48/-1	61/60/-1	42/43/1
Cheyne–Stokes respiration	52/53/1	48/49/1	46/45/-1	56/55/-1

**Table 8:** The average and standard deviation of the short-term energy of the 5 respiratory patterns (part data).

Respiratory patterns	Short-term energy average/standard deviation			
Normal respiration	8.34/5.16	18.64/7.02	8.39/6.31	8.41/6.21
Biot's respiration	11.99/7.99	11.55/7.61	9.67/10.61	6.29/5.92
Tachypnea	10.63/8.37	13.31/8.18	8.41/4.78	11.26/7.09
Bradypnea	9.20/5.47	15.16/8.85	9.34/6.92	12.94/7.62
Cheyne–Stokes respiration	6.06/5.94	9.20/8.06	3.71/6.23	7.18/7.46

**Table 9:** The average, standard deviation, and minimum of the instantaneous frequencies of the 5 respiratory patterns (part data).

Respiratory patterns	Average	Standard deviation	Minimum
Normal respiration	0.16	0.11	0.02
	0.31	0.10	0.10
	0.50	0.34	0.01
	0.29	0.18	0.04

Biot's respiration	0.54	0.34	0.00
	0.11	0.09	0.00
	0.19	0.14	0.00
	0.30	0.25	0.00

Tachypnea	0.55	0.33	0.02
	0.62	0.32	0.02
	0.57	0.29	0.01
	0.68	0.34	0.02

Bradypnea	0.49	0.26	0.01
	0.42	0.21	0.01
	0.40	0.26	0.01
	0.51	0.27	0.01

Cheyne–Stokes respiration	0.36	0.28	0.00
	0.48	0.34	0.00
	0.38	0.42	0.00
	0.35	0.29	0.00

**Table 10:** The experimental results of the 10-fold cross-validation method.

Times	1	2	3	4	5
SVM (%)	100.00	97.50	95.00	98.75	98.75
KNN (%)	90.00	88.75	88.75	88.75	90.00
Times	6	7	8	9	10
SVM (%)	98.75	97.50	98.75	95.00	98.75
KNN (%)	91.25	90.00	88.75	90.00	87.50

**Table 11:** The classification results of different classifiers.

Classifier	Accuracy (%)	Cohen kappa score	Classification label
SVM	98.25	0.978125	1/2/3/4/5
KNN	88.75	0.859375	1/2/3/4/5

## Data Availability

The data used to support the findings of this study are included within the article.
